RETRACTED

# Complete Lumbar Spine Dislocation With Full Neurological Recovery

**DOI:** 10.7759/cureus.19249

**Published:** 2021-11-04

**Authors:** Abdulaziz M Alshamrani, Ahmed M Aldawsari, Saud A Alhassoun, Abdulrahman M Albahkali, Nawaf F Alhussain, Abdulaziz L Moqeem, Reem H Mohammed, Anhar M Hasanain, Afnan M Almutairi, Haider M Abu Shaheen, Abdullah A Al Qarni, Ali A Al Khalaf, Khalifah K Alfarhan, Fawaz M Alzubaidi, Malak Alshammari

**Affiliations:** 1 College of Medicine, Prince Sattam Bin Abdulaziz University, Al-Kharj, SAU; 2 College of Medicine, Imam Mohammad Ibn Saud Islamic University, Riyadh, SAU; 3 College of Medicine, King Saud Bin Abdulaziz University For Health Sciences, Riyadh, SAU; 4 Family Medicine, Directorate of Health Affairs, Jeddah, SAU; 5 College of Medicine, Ibnsina National College, Jeddah, SAU; 6 College of Medicine, King Abdulaziz University, Jeddah, SAU; 7 College of Medicine, Tabuk University, Tabuk, SAU; 8 College of Medicine, Imam Abdulrahman Bin Faisal University, Dammam, SAU; 9 College of Medicine, King Khalid University, Abha, SAU; 10 College of Medicine, King Faisal University, Hofuf, SAU; 11 College of Medicine, Umm Al Qura University, Mecca, SAU

**Keywords:** vertebral facture, case report, fall from height, fracture-dislocation, lumbar spine surgery

## Abstract

The thoracolumbar region is the most vulnerable segment of the spine to traumatic injuries. It represents a region of transition of the relatively fixed and immobile thoracic spine and flexible lumbar spine. Injuries to the thoracolumbar region often result from high-energy trauma. We present the case of a 24-year-old woman who was brought to the emergency department after a fall from a great height. She presented with severe back pain that was associated with the inability to move both of her lower limbs with absent sensation and loss of urinary and bowel continence. Otherwise, she was hemodynamically stable. The patient underwent a computed tomography scan of the abdomen and pelvis. It demonstrated a complete fracture-dislocation of the second lumbar vertebra relative to the first lumbar vertebra causing shortening of the vertebral column. The second lumbar vertebra had a complete lateral dislocation and appeared in the same axial plane as the first lumbar vertebra giving the appearance of a “double vertebrae” sign. The patient was prepared for emergency open reduction internal fixation with a posterior surgical approach. The operation was done under general anesthesia with the use of sensory-evoked potential responses to avoid any neurological injury. Good realignment of the thoracolumbar spine was achieved. Six months after the operation, the patient was asymptomatic and resumed her regular activities. Complete traumatic lateral dislocation of the lumbar spine is very rare. Early diagnosis of such fracture by computed tomography scan is crucial to avoid maneuvers that may cause unintended spinal cord injuries.

RETRACTED

## Introduction

The thoracolumbar region is the most vulnerable segment of the spine to traumatic injuries. It represents a region of transition of the relatively fixed and immobile thoracic spine and flexible lumbar spine. Injuries to the thoracolumbar region often result from high-energy trauma. These include falls from heights, road traffic accidents, extreme sports activities, and work-related injuries [1]. It is estimated that up to 25% of patients who sustained high-velocity spine trauma develop spinal cord injury [2]. However, fracture-dislocation of the thoracolumbar spine is rare and accounts for less than 3% of all vertebral column fractures [1]. A thoracolumbar spinal injury can result in severe and disabling neurological with devastating effects on the patient’s quality of life. Here, we report the case of a young woman with complete traumatic lateral dislocation who had a complete neurological recovery, which is extremely rare with few similar reported cases in the literature [3].

## Case presentation

We present the case of a 24-year-old woman who was brought to the emergency department 30 minutes after a fall from height. She had an accidental fall from her home roof of three stories. She presented with severe back pain that was associated with the inability to move both of her lower limbs with absent sensation. Further, the patient had complete urinary and bowel incontinence.

On examination, the patient appeared in significant pain and distress. She had extensive abrasions over her lower limbs. Her vital signs were a pulse rate of 130 bpm, blood pressure of 125/74 mmHg, respiratory rate of 15 bpm, and temperature of 37.2℃. The patient was alert, conscious, and oriented. His Glasgow Coma Scale was 15/15. Neurological examination revealed hypotonia and power of 0/5 in both proximal and distal muscle groups of the lower limb. The patient had lost touch and pain sensation in both lower limbs. Palpation of the lumbar spine revealed severe tenderness on palpation with step-like deformity. The knee and ankle jerk reflexes were absent. The anal tone was absent. Initial laboratory investigations were within the normal limits (Table 1).

**Table 1:** Summary of the results of laboratory findings

Laboratory Investigation	Unit	Result	Reference Range
Hemoglobin	g/dL	14.8	13.0–18.0
White Blood Cell	1,000/mL	4.5	4.0–11.0
Platelet	1,000/mL	350	140–450
Erythrocyte Sedimentation Rate	mm/hr	10	0–20
C-Reactive Protein	mg/dL	4.2	0.3–10.0
Total Bilirubin	mg/dL	0.8	0.2–1.2
Albumin	g/dL	4.5	3.4–5.0
Alkaline Phosphatase	U/L	36	46–116
Gamma-glutamyltransferase	U/L	40	15–85
Alanine Transferase	U/L	53	14–63
Aspartate Transferase	U/L	28	15–37
Blood Urea Nitrogen	mg/dL	8	7–18
Creatinine	mg/dL	0.8	0.7–1.3
Sodium	mEq/L	138	136–145
Potassium	mEq/L	4.0	3.5–5.1
Chloride	mEq/L	105	98–107

The patient underwent a computed tomography scan of the abdomen and pelvis. It demonstrated a complete fracture-dislocation of the second lumbar vertebra relative to the first lumbar vertebra causing shortening of the vertebral column. The second lumbar vertebra had a complete lateral dislocation and appeared in the same axial plane as the first lumbar vertebra, giving the appearance of a “double vertebrae” sign. The posterior elements of both the first and second vertebrae were fractured and were separated from their vertebral bodies resulting in widening of the vertebral canal (Figures 1, 2). There was no evidence of hemoperitoneum. The internal organs appeared unremarkable with no injuries. No other fractures were observed.

RETRACTED

**Figure 1:** Coronal computed tomography image of the spine demonstrating complete lateral dislocation of the lumbar spine (arrow)

**Figure 2:** Axial computed tomography image demonstrating both the first (long arrow) and the second (short arrow) lumbar vertebrae at the same axial plane

Since the patient was hemodynamically stable, she was prepared for emergency open reduction internal fixation with a posterior surgical approach. The operation was done under general anesthesia with the use of sensory-evoked potential responses to avoid any neurological injury. A midline thoracolumbar incision was made. The paravertebral muscles were severely injured. Laminectomy was performed for the second lumbar vertebra. The dura was found intact. Vertebral column restoration was performed by long segment fixation. Good realignment of the thoracolumbar spine was achieved. The patient tolerated the procedure well with no neurological injury noted by the monitor. She underwent an intensive physiotherapy rehabilitation program. Six months later, the patient was asymptomatic and resumed her regular activities. She had full power of both lower limbs with urinary and bowel control.

## Discussion

We presented the case of a young woman with complete lateral lumbar dislocation with complete neurological recovery. Very few cases reported in the literature had neurological recovery after such severe spinal fracture. As in the present case, fracture of the pedicles was involved in all the reported cases with neurological improvement. It is postulated that the separation of the posterior element of the vertebral bodies provides enough space to avoid injury to the spinal column by spontaneous decompression [4].

RETRACTED

Complete traumatic dislocation of the spinal cord is very uncommon and is rarely seen in clinical practice. The majority of patients have co-existing organ injuries and may die from hypovolemic shock at the scene. Further, such fracture can cause transection of the spinal cord. Neurological recovery after such fracture-dislocation is very unusual [5]. A literature review by Zeng et al. [3] in 2018 showed that only six cases were reported in the literature with complete fracture-dislocation of the thoracolumbar spine had a good outcome.

It is of paramount importance to establish the diagnosis of spinal fractures early. Such fractures may be evident on plain radiographs. However, computed tomography scans can provide an accurate assessment of vertebral column injuries. The scan may demonstrate the “double vertebrae” sign, in which two vertebrae are seen at the same axial level. Early diagnosis prevents improper maneuvers that may precipitate spinal cord injury resulting in further neurological deficits [6].

Surgical treatment is advised for all cases of fracture-dislocation of the thoracolumbar spine [7]. The posterior surgical approach is recommended considering the severe instability of the injured spine. The goal of the treatment is to achieve realignment and fixation to prevent any neurological injuries. The time of surgery, however, is controversial [8]. In the present case, the surgery was conducted within 24 hours as the patient was hemodynamically stable and had no other associated injuries.

## Conclusions

Complete lateral dislocation of the thoracolumbar spine is very rare. Clinicians should have a high index of suspicion for spinal fractures in any patient with high-energy trauma and should request a computed tomography scan for an accurate evaluation of the spinal cord. Early diagnosis of spinal fractures prevents unintended neurological injuries resulting from inappropriate maneuvers. While complete lateral dislocation of the lumbar spine often results in transection of the cord with paraplegia, the present case demonstrated the possibility of complete neurological recovery. In patients with hemodynamic stability, surgical restoration with long fixations should be performed with no delays for patients with complete traumatic lumbar dislocations.
